This article has been retracted.

# An Efficient and Reliable Routing Method for Hybrid Mobile Ad Hoc Networks Using Deep Reinforcement Learning

**DOI:** 10.1155/2020/8888904

**Published:** 2020-12-11

**Authors:** Murtadha M. A. Alkadhmi, Osman N. Uçan, Muhammad Ilyas

**Affiliations:** ALTINBAŞ University, Engineering and Naturel Science, Mahmutbey, Istanbul, Turkey

## Abstract

With the reliance of humans on mobile smart devices that have wireless communication, modules have significantly increased in recent years. Using these devices to communicate with the survivors during a disaster or its aftermath can significantly increase the chances of locating and saving them. Accordingly, a method is proposed in this study to extend the lifetime of the nodes in a Mobile Ad Hoc Network (MANET) while maintaining communications with the nearest base station (BS). Such a methodology allows the rapid establishment of temporary communications with these survivors, as restoring the complex infrastructure is a time-consuming process. The proposed method achieves the longer lifetime of the network by balancing the load throughout the nodes and avoids exhausting those with limited remaining energy. The proposed method has shown significant improvement in the lifetime of the MANET while maintaining similar Packet Delivery Rate (PDR) and route generation time, compared to existing methods.

## 1. Introduction

Reliance on smart mobile devices, such as smartphones and tablets, has rapidly increased in recent years, according to the enormous number of services that are being provided through these devices, besides traditional communication services [1–3]. These devices are mainly connected to two types of wireless networks, a cellular network that provides basic communication services, such as phone calls, messaging, and internet, and Wi-Fi networks, which provide much less-expensive internet, compared to cellular data [4–6]. Providing these networks requires intense infrastructure to connect these devices to the other parts of the networks and the internet. This infrastructure provides an access point, i.e., base station (BS), for each device to connect it to the remaining parts of the network and other networks [7].

Such infrastructures can suffer from severe damages when a disaster, such as wars, natural disaster, and terrorist attacks, occurs. Reestablishing these networks is a time-consuming process, according to the complexity and intensity of the required infrastructure to reestablish communications. Moreover, the importance of these communications during such a disaster, or during the aftermath, is significant to establish communications with any survivors or those in need of assistance. Thus, a wireless ad hoc network (WANET) can be established by using the same devices as nodes to deliver the data packets to the nearest online BS. Moreover, as these devices are hand-held and according to the high possibility that the owners of these devices are on the move, to escape the disastrous area, Mobile Ad Hoc Network (MANET) is more suitable to such a scenario [8, 9].

With the absence of the infrastructure and the use of mobile nodes to route the packets, finding the optimal route has raised as an emerging problem. Several studies have used overlay network technology [10–12] to route the packets in a hybrid network that uses MANET to establish communications with a base station. These methods are presented as improvements to the standard protocols with the aim of preventing crashing in these networks. However, these methods mainly are aimed at optimizing energy consumption [13, 14] or focusing on three-layered routing to optimize the packet flow by reducing the routing overhead [15–18]. Recently, a Software Defined Network (SDN) has attracted significant attention in optimizing the routing in such networks [19–23].

Naser and Kadhim [19] present three SDN-based routing methods for MANETs. The aim of the proposed method is to reduce the power consumption in the network by minimizing the routes the data travel through, in a clustered MANET. However, despite the relatively improved network lifetime, emphasizing on reducing power consumption can exhaust the resources available on certain nodes. If such nodes are located in key-positions, in which a lot of traffic is routed through these nodes to shorten their paths, these nodes can die significantly faster than when the loading is distributed on multiple nodes. Using slightly longer paths to reduce the loading on certain nodes can maintain a larger number of nodes alive for a longer time, despite the possibility of increasing the end to end (E2E) delay of packets. However, extending the lifetime of each and every node in the MANET is a very important aspect in disastrous scenarios, as these nodes are used to establish communications with their owners.

In addition to the extension of the lifetime of the nodes in the MANET when the loading is distributed among the nodes, the results of the experiments conducted by Poularakis et al. [24] show that the use of backup paths has been able to improve the performance of the networks. Poularakis et al. [24] propose a hybrid routing method that allows the SDN controller to define the routes but also allows the nodes to make their own decision whether to follow that route or adapt to the current state of the network. This method is intended to be used by tactical networks, in which communications among the devices at a certain geographical area are more intense than those with squads in other areas. Hence, this method is aimed at maintaining communications within reachable devices even if the communications with the SDN are no longer available. However, in a disastrous scenario, communications among isolated devices are useless, unless one of these devices can reach a BS to deliver the messages.

The method proposed by Lee [8] uses deep learning to classify the node degree in order to assign virtual routes. This method is proposed to establish communications among MANET nodes in ad hoc topology to establish communications with the nearest BS during a disaster. Accordingly, this method considers the connectivity of the nodes as the utmost important factor. However, this method does not take the energy remaining at each node into consideration when producing the routes. Hence, it is possible that this method assigns a route through a node with very low remaining energy despite the ability to use another route that can avoid exhausting this node. Moreover, this method supposes a limited movement speed of the node (0-3 km/h), which may not be the case when people are escaping certain disasters. The speed limitation is according to the use of a feed-forward neural network in the classification task, which cannot take into consideration historical data that can accurately represent the movement of the nodes.

Kadam and Srivastava [25] proposed a routing method for wireless sensor networks (WSNs) based on Q-learning, i.e., reinforcement learning. This method takes into consideration the energy remaining at each node and has been able to significantly improve the lifetime of the network, by avoiding the use of nodes with low remaining energy in routing packets, as long as alternative routes exist. However, the nodes in the WSN are considered static in this method, so that it cannot be applied in MANETs. Moreover, this routing method requires each node to make a decision for each incoming packet, based on its destination, which can in return be a power-consuming task. However, as the data in WSNs may flow from one node to another; i.e., there is no sink node that collects all data; maintaining a routing table is important for each node.

Based on this review, the methods that exist in the literature have addressed the problem of establishing temporary communications using MANETs, even by using deep learning [8] and reinforcement learning [25]. However, these methods can handle networks with limited speed of nodes, which may be a dramatic limitation to these methods as survivors tend to flee the location of a disaster as fast as possible. Moreover, despite the ability of certain methods [19, 24] to minimize the power consumption of MANETs by using the shortest possible paths, such aim can exhaust certain nodes in the MANET, which can affect the lifetime of these nodes, despite the extension of the network's lifetime. Thus, in order to maximize the chances to locate and save survivors, it is important to extend the lifetime of the MANET, taking into consideration maximizing the lifetime of each individual node in the network.

In this paper, we proposed a new SDN-based routing method for MANETs. The proposed method is aimed at providing temporary communications to devices in a disastrous area, during the disaster of the aftermath. The established temporary network uses ad hoc topology, in which each node may act as a hop in the route to deliver a certain packet initiated from another node. Mainly, the proposed method is aimed at extending the lifetime of the nodes in the network for the maximum possible lifetime by avoiding exhausting the resources of certain devices as long as alternative routes are available, in addition to emphasizing the connectivity of each node. The use of alternative routes also allows multiple sources to communicate with the BS simultaneously, as no bottleneck nodes exist in the network. Moreover, the proposed method takes into consideration the movement of the nodes in the area, regardless of their speed. Such a consideration can be achieved by collecting and using historical data, which allows predicting the future position of the node based on its speed and trajectory.

## 2. Materials and Methods

### 2.1. Overview of the Proposed Method

The proposed method requires the existence of a BS that can handle all the required applications to the devices in the network. Then, the devices in the disastrous area act as nodes to create a MANET, in which all devices aimed at connecting to the BS, which makes it the sink node. In case that all the nodes are out of the range of the BS, an additional node can be positioned in the region to close such a gap. However, the proposed method considers that a virtual connection exists between the BS from one side and each device from another, directly or through one or more nodes. This requirement is based on the fact that all devices must connect to the service provider in order to deliver their messages. Local networks that cannot reach BS have no importance as the devices in these networks cannot deliver their messages to the service provider. Hence, a dedicated server can be located at the BS side, as all BSs are already connected to each other using the infrastructure built prior to the disaster, in order to communicate with the nodes, collect their information, and control the packets flow in the network, as shown in Figure 1.

### 2.2. Network Initialization

Initially, the proposed method collects information about the nodes in the MANET in order to produce the optimal routes for each node to establish communications with the BS. This discovery uses a reverse-routing approach, which is an inefficient routing method that relies on reversing the path that a packet travels from the BS to the node. First, a “Hello” packet is sent from the BS to all the nodes that are within its range. Each node then forwards the packet to all adjacent nodes, i.e., within its range. If the packet is received by a node that already has received it from another node, the packet is dropped. Otherwise, the node sends an acknowledgment to the node that delivered the packet and appends its ID to the packet and forwards it to the nodes within its range. If the node receives an acknowledgment from the nodes is has sent the packet to, it waits for a response from that node, as the node has received the Hello packet but still discovering further nodes. Otherwise, the node sends back its position, range, and remaining energy (percentage) to the node that delivered the Hello packet. This node appends the data received from all the nodes that have acknowledged the arrival of the hello packet and adds its own information then sends it to the node the delivered Hello packet. This process is repeated until all the nodes' information is delivered to the BS, as shown in Figure 2.

### 2.3. Deep Reinforcement Learning

The main aim of reinforcement learning (RL) is to recognize the outcome of each action an agent can execute in a certain environment, based on the state of the agent in that environment [26]. Theoretically, the agent attempts all possible actions per each possible state in the environment, so that the action that produces the best outcome is executed during the runtime of the agent. However, especially in complex environments, it is impossible to replicate all the possible states during the training of the agent. Thus, an approximation function is required to predict the outcome of each action based on the state of the agent, so that even the outcome of the possible actions for states that the agent has not been through during the training can be predicted based on similar states that the agent has been through.

According to the outstanding performance of artificial neural networks in approximating complex functions, these networks are being used by RL agents to solve the problem of predicting outcomes of the possible actions for a certain state that is not included in the training. The state of the agent is fed to the neural network, and the outcome, denoted as *Q*, of each action is collected from the output. During the training, the reward that represents how good the response of the environment is for a certain action is used to train the neural network, by assigning this value to the neuron correspondent to the selected action. As the neural network has no initial knowledge about the environment, random actions are executed and used to train the neural network. As more knowledge is gained, the selected actions start to rely on the predictions of the neural network, by selecting the action that the neural network predicts to have the highest reward, i.e., *Q*, value. The selection of the action, random or based on the neural network, is governed by a value, denoted as epsilon, that starts with a high value and is reduced as the neural network gains more knowledge. A random number generated and compared to the epsilon and a random action is selected if the random number is less than epsilon; otherwise, the action that has the highest *Q* value from the neural network is selected.

In some applications, such as routing, the outcome of an action cannot be recognized immediately. Alternatively, a series of actions must be conducted before evaluating the response of the environment, i.e., whether the packet is delivered or not. Thus, in such a scenario, the training of the neural network is postponed until all the required actions are executed and a reward is provided by the environment. Then, depending on the importance of each action, based on its position in the series, the reward value is discounted using a discount factor and used to train the executed action at the state it is executed in. A higher discount factor, close to one, indicates that the position of the action has less importance; i.e., earlier actions can have the same influence on the outcome as the recent ones. Such a high value is suitable for the required application, i.e., routing packets in MANET, as the selection of each hop can have equal influence on the selected route.

Traditionally, a Deep Q-Network (DQN) is used to predict the *Q* value of each action at a certain state, which represents the reward value expected from the environment at that state if the corresponding action is selected. Further improvement to the performance of RL is proposed by branching the last hidden layer into a group of neurons, equal to the number of possible actions, and a single neuron [27], as shown in Figure 3. Then, the output layer adds the value outputted by the single neuron, which represents the quality of the state the agent is currently at, to each value in the action group of neurons. Hence, the number of neurons in the output layer is equal to the number of actions and the outputted values also represent the *Q* value per each action. However, the use of the average of *Q* values to describe the state of the agent can be beneficial to evaluate being in that state, as overall, as well as the ability to evaluate each action whether to improve the state of the agent or worsen it. Thus, better training can be provided to the neural network, which also improves the predictions collected from it during runtime.

Several types of neural networks exist, which have shown different capabilities of processing different types of inputs. For instance, if each input is characterized using a one-dimensional feature vector, fully connected; i.e., dense, neural networks have shown good performance processing such inputs, in terms of complexity and quality of predictions. Recurrent Neural Networks (RNN) have shown better performance handling time-series data, in which the positions of the values influence the characteristics of the input. Moreover, Convolutional Neural Networks (CNN) have shown significantly better performance in processing three- and four-dimensional inputs, such as images. This type of neural networks convolutes two- or three-dimensional filters over the input to detect multidimensional features, based on the number of dimensions of the filters.

### 2.4. MANET Representation and Neural Network Implementation

An accurate and efficient representation of the environment to the agent can significantly improve its performance, by providing accurate predictions rapidly. Accordingly, only information relative to the routing task is collected from each node, which is sent by the node in a reply to the “Hello” message that is sent by the BS during the network initialization. The data required from each node are as follows:

- The position of the device: all modern devices are equipped with a positioning system, mostly based on the Global Positioning System (GPS), which can provide the coordinates of the device with high accuracy.
- The remaining energy: all smart devices measure and display the percentage of the energy remaining in their energy sources, mostly batteries. This value is also sent to the BS in percentage.
- Range: this is the distance that the wireless module on the device can achieve, as these devices are equipped with different communication modules that can achieve different ranges.

As the nodes in the MANET are moving, the position can change over time and the faster the node is moving the more change in position is detected in a fixed time window. Moreover, the remaining energy can also be changing over time, mainly decreasing, as the device is being used. Thus, it is important to represent the changes in these two values to the implemented neural network. However, to maintain efficient representation, i.e., to avoid providing huge data that require intensive processing, a single array is used to represent both changes. This array has dimensions of 512 × 512 × 3. The last three energy measurements are mapped according to the position of the node at the time the energy is measured, as shown in Figure 4, which shows that the neural network can detect the movement of the node *N*_1_, as well as the change in its remaining energy.

Another array is also used as the input of the neural network, which represents the current position of the nodes in the MANET. To emphasize these positions and allow the neural network to exploit this input at several levels, and all the values in this array are set to zero, except the mapped positions of the nodes in the network, which are set to ones. Hence, this layer has 512 × 512 × 1 dimensions. Another array is created to represent the range that each node can reach, mapped to the 512 × 512 dimension. This array is also filled with zeros before setting a circle filled with ones around each node, based on its mapped range. Thus, the ranges of nodes that can communicate with each other interfere as shown in Figure 5.

Additionally, three arrays are created, each has a dimension of 512 × 512 × 1 and all are filled with zeros except the position of the source node in the first array, the position of the BSs, i.e. sink nodes, in the second layer and the position of the node that the packet is currently at, as the proposed method predicts the next-hop once per each prediction. Finally, an array is created and the ratio between the numbers of routes that pass through each node to the total number of nodes is calculated, up to the current routing step.  Figure 6 summarizes these three arrays for the current routing task of the sample MANET shown in the same figure.

Inspired by the U-net neural network [28], the neural network implemented for the proposed method uses a similar approach, in which the input of the neural network and the outputs of certain layers are appended to the inputs of the layers closer to the output layer, as shown in Figure 7. This approach allows the proposed neural network to consider the characteristics of the MANET, especially the exact positions of the nodes, in the outputted values.

The neural network that is implemented for the proposed method consists of three main parts. The first part processes the 512 × 512 × 3 array that represents the energy change in energy and position, extracts the required features, and produces a 512 × 512 × 1 array, as shown in Figure 8. Two convolutional layers, one two-dimensional and one three-dimensional layers are used, where the three-dimensional layer uses a filter with a size of 1 × 1 × 64 to summarize the 64 features detected by the 64 two-dimensional filters to produce the required shape. The outputted array is then concatenated with the remaining inputs to produce a single 512 × 512 × 6 array.

The output of the concatenation layer is then processed by a CNN similar to the structure of the standard U-net but uses the “same” padding techniques, in which the dimension of the output array is identical to the input one. Such output is achieved by padding the image with additional zeros, i.e., extending the dimension of the input array, according to the size of the filters in the convolutional layer.  Figure 9 summarizes the structure of the implemented neural network.

The output of this part of the neural network is then forwarded to the network shown in Figure 10. The output of this part, which is the output of the entire neural network, consists of two components, a two-dimensional array “Hop” and a single value “State.” The value outputted by the “State” neuron represents the overall quality of the agent when being at that state. For instance, packets currently in nodes closer to the BS are expected to have higher “State” value. Moreover, the values in the output of the “Hop” layer represent the advantage of forwarding the packet to any position in the region. However, according to the use of the positions array in the input and by considering avoiding outputting values at positions that do not contain a node, the output that has the maximum value is expected to be located on a position of a node. Nevertheless, the proposed method selects the node closest to the position that has the highest output to forward the packet to.

### 2.5. Training the CNN and Routing the MANET

As illustrated earlier, RL has the ability to postpone the training process until all the required actions are executed and a reward value can be calculated. Thus, the proposed neural network is used to route the packets and then a reward is calculated based on the performance of the MANET using the selected routes. To define the route that the packets must follow from a certain node to the BS, the information received with the “Hello” message is fed to the neural network. Initially, the position of the value one in the array that represents the current hop the packet is at is identical to the array that represents the source packet. The position of the node nearest to the maximum value in the output of the Hop layer is then selected as the next hop. The position of the value one is then mapped according to the newly selected node and fed to the neural network until a node that is directly connected to the BS is reached. When the route is defined, the information is sent to each node involved in the selected path, indicating that any packet incoming from the source node must be forwarded to the designated node.

When a node loses connection to one of the other nodes that exist in its routing table, this node instantly sends the same set of information to the nearest node that also exists in its routing table, which is used to route packets incoming from other nodes. If such a node does not exist, it sends the information to the nearest available node, in order to update the BS with the new position and to request a new route. Additionally, the proposed method also sends periodic “Hello” messages in order to discover any newly connected devices and update the positions of the existing nodes. This allows updating and producing the required 512 × 512 × 3 array that reflects the changes in the energy and position.

When a node is selected based on the predictions of the neural network, the selection is validated against the path defined so far. If the node is found to exist in the path, the neural network is trained immediately with a reward value of -1, i.e., a punishment, and a new prediction is collected. This ensured avoiding producing loops in the network, which can dramatically reduce the performance of the network. As the aim of the proposed method is to extend the lifetime of each device in the network and maintain their connectivity, the reward value is calculated based on these factors, as shown in Equation (1). The exact same network is routed using the standard Ad hoc On-Demand Distance Vector (AODV) protocol, and the performance of the MANET is measured based on the lifetime of the device that dies first and the Packet Delivery Rate (PDR). According to the formula, a reward of one is used to train the neural network if it achieved identical performance to the use of AODV. Any additional improvement in the performance increases the reward value, while any lower performance reduces the reward value. Accordingly, the proposed method learns to improve the overall performance of the MANET, without emphasizing one factor over the other, which is the reason behind multiplying each performance measure by the other from the AODV-based performance.

(1) $$\begin{array}{c} R=\frac{L_{\text{AODV}}\times \text{PD}{\text{R}}_{\text{RL}}+L_{\text{RL}}\times \text{PD}{\text{R}}_{\text{AODV}}}{L_{\text{AODV}}\times \text{PD}{\text{R}}_{\text{AODV}}}, \end{array}$$

where the *L*_AODV_ and PDR_AODV_ are the lifetime and PDR of the AODV-based MANET and *L*_RL_ and PDR_RL_ are the lifetime and PDR for the MANET using the proposed RL-based routing method.

## 3. Results and Discussion

A model is implemented for the proposed method using Python programming language, in which the Tensorflow library is used to implement and operate the neural network. The Sim2Net (https://pypi.org/project/sim2net/) library is used to simulate the wireless sensor networks and interact with the proposed model that is responsible for routing the packets in the network. This implementation allows direct interaction between the simulated wireless network and the implemented rout selection model; i.e., the node vectors are directly collected from the network and processed by the model, in order to recognize the optimal route. Mainly, the performance of the proposed method is validated by comparing the performance of the network when the proposed method and three of the standard and widely used routing protocols in MANETs are used. These protocols are the Ad hoc On-Demand Distance Vector (AODV) [29], Optimized Link State Routing (OSLR) [30], and Zone Routing Protocol (ZRP) [31]. The main parameters of the simulated network are shown in Table 1.

### 3.1. Packet Delivery Rate (PDR)

As illustrated in the experimental setup, the performance of the proposed method is evaluated using fifteen different scenarios, according to the existence of three numbers of mobile nodes and five numbers of base stations; i.e., per each number of base stations, the three numbers of mobile nodes are evaluated. Per each scenario, the ratio between the numbers of packets that are delivered to the base stations to the total number of packets initiated by the mobile nodes is measured for the proposed method, as shown in Figure 11. These results show that the proposed method has been able to maintain similar performance when the network has a high density of nodes. Such behavior is according to the existence of several alternative routes that the proposed method can use to deliver the packet. Additionally, the probability of delivering a packet is also increased when the number of base stations in the region is increased. The existence of these stations also allows more flexibility to deliver the packet, by providing more possible routes.

### 3.2. Route Discovery Time

As each node waits for the remaining nodes that are in its range and have not received the “Hello” message from the base station to discover their network and reply back to that node, the arrival of the nodes vectors from a certain node indicates that all the network behind that node is discovered. Accordingly, when the base station receives the node vectors from all the nodes that are directly connected to it, network discovery can be considered complete and the routing table generation process can be initiated. As shown in Figure 12, in addition to the lower time required by the proposed method to discover and assign a route to each node in the network, the relation between the time and number of nodes is almost linear and irrelative to the number of base stations. Such a relationship is according to the fact that the input to the neural network contains all the information of the network, so that the neural network requires no additional processing if an additional base station exists. However, as increasing the number of nodes in the network increases the number of routes to be discovered, the proposed method requires additional time to discover these routes. Similar behavior is noticed in the OLSRv2 protocol, despite the significantly higher discovery time, which is the highest among all protocols.

In contrast, the time required by the AODV protocol to discover the routes is exponentially dependent on the number of nodes in the network and the number of base stations. Such an increase in time is according to the need for route discovery per every query, so that more computations are required when more nodes exist in the network, according to the additional traffic generated by the nodes. Similarly, the number of zones is also increased when the number of nodes is increased while using the ZRP. Hence, the time required to discover the routes increases significantly when additional nodes are added to the network. Thus, in terms of route discovery time, the proposed method has been able to achieve significantly better performance, especially by maintaining similar times even when the number of base stations is increased; i.e., more possible routes exist in the network.

### 3.3. Network Lifetime

Extending the lifetime of each node in the network is the main aim of the proposed method, according to the significant importance of this extension to maintain communications during or after the disaster for as long as possible. Accordingly, this experiment evaluates the lifetime of these devices by monitoring the energy of each node. When the energy of one of the nodes becomes less than the energy required to transmit a data packet, the node is considered dead. The lifetime of the network is measured between the initialization of the network and the loss of the first node. Accordingly, the simulation is not governed by any interval and continued until one of the nodes exhausts all its energy. As shown in Figure 13, the proposed method has been able to extend the lifetime of the nodes, which indicates that the loading has been balanced among the nodes, to avoid exhausting the resources of certain nodes. However, the gap between the lifetimes of the networks with different numbers of nodes is larger at a lower number of base stations. The lack of alternative routes in such cases is the main reason behind forcing the proposed method to exhaust certain nodes that are in the route of the base stations to deliver the packets. Providing alternative routes, by increasing the number of nodes or base stations, has been able to significantly improve the performance of the network when using the proposed routing method.

## 4. Conclusions

Establishing communications during a disaster or the aftermath is a vital feature to locate and save any survivors. However, during such a disaster, the infrastructure that is required to establish wireless communications, such as cellular, is most probably affected by a disaster. The establishment of such an infrastructure is a time-consuming process, which cannot normally be accomplished during the search and rescue operations. Thus, MANETs are being used to establish temporary communications with the survivors, through their everyday digital devices. With the limited energy available in these devices and the need for those devices to route the packets to the BS, it is important to improve the efficiency of energy usage, so that the overall lifetime of the MANET as well as the lifetime of each node is extended to maximum, to improve the chances of locating and saving the survivors.

A new routing method is proposed in this paper to efficiently connect the nodes in a MANET to an operating BS to establish communications with survivors during the occurrence or the aftermath of a disaster. The proposed method is aimed at increasing the lifetime of the network by balancing the loading on the nodes and avoiding exhausting the ones with limited remaining energy. This aim is achieved by using RL, in which a neural network considers the status of the network to predict the route for a node to the BS. The use of the proposed method can extend the lifetime of the devices, which can significantly increase the chances of saving lives. In addition to the better lifetime, the proposed method has been able to achieve similar performance, compared to existing routing protocols, in terms of the PDR and route discovery time. Moreover, as the nodes in the wireless network are mobile with relatively high speeds, the proposed method can provide efficient communications to the search and rescue teams during the search for and extraction of survivors.

In a future work, the ability to use Generative Adversarial Networks (GANs) to generate the route directly based on the inputted state of the MANET is according to the ability of these neural networks in producing complex multidimensional output. The routes that are going to be used to train the neural network are going to be generated using the method proposed in this study. Hence, the same routes can be generated while significantly reducing the route generation time.

## Figures and Tables

**Figure 1:** A sample hybrid wireless ad hoc network.

**Figure 2:** Propagation of the “Hello” packet and replies from the nodes.

**Figure 3:** DQN and dueling Q-Network: (a) traditional DQN and (b) improved dueling Q-Network [27].

**Figure 4:** Sample slices of the 512 × 512 × 3 energy array, which shows the rate of change in the remaining energy and the movement of the node.

**Figure 5:** Illustration of the array that represents the ranges of the nodes.

**Figure 6:** Positioning of the source node, base stations, and the node that the packet is currently at.

**Figure 7:** Structure of the U-net [28].

**Figure 8:** Processing of the energy array and concatenation with the remaining inputs.

**Figure 9:** Structure of the part of the implemented CNN similar to the U-net.

**Figure 10:** Processing the output of the U-net-similar part to achieve dueling Q-learning.

**Figure 11:** PDR versus the number of base stations in the region.

**Figure 12:** Influence of the number of base stations and mobile nodes on the route discovery time.

**Figure 13:** Lifetime of the wireless network versus the number of base stations.

**Table 1:** Parameters of the experimental setup.

Parameter (unit)	Value
Simulation time (sec)	300
Pause time (sec)	60
Data type	Constant Bit Rate (CBR)
Size of each packet (byte)	512
Network area (m^2^)	3000 × 3000
Range of each node (m)	MN: 375, BS: 375
Number of nodes	MN: [50, 100, 150], BS: [1–5]
Energy (joule)	MN: 1, BS: unlimited
Packet transmission energy (joule)	5 × 10^−9^
Nodes movement	Random walk
Maximum node speed (km/h)	10

## Data Availability

There have been no data collected during this study. All evluation was conducted by simulating the networks. Hence, the same simulation environment can be replicated based on the parameters described in the paper.
